RETRACTED

# Optimal Defect Detection and Sensing System of Railway Tunnel Radar considering Multisensor System Combined with Active Interference Suppression Algorithm

**DOI:** 10.1155/2022/2459996

**Published:** 2022-04-25

**Authors:** Yang Lei, Yong Zou, Bo Jiang, Tian Tian

**Affiliations:** ^1^China Academy of Railway Sciences, Beijing 100081, China; ^2^Beijing ZhuoRuiXinDa Technology Co., Ltd, Beijing 101599, China

## Abstract

With the rapid development of science and technology, testing equipment and testing methods are constantly updated. Radar detectors have the advantages of losslessness, high efficiency, high resolution, and high-speed radar image capture. They can accurately locate defects in railway tunnels, respond to hidden dangers in time, and provide strong technical support for transportation. This paper proposes to optimize the defect detection of railway tunnel radar through the combination of multisensor technology and active interference suppression algorithm and designs the corresponding sensor system according to the content. This article analyzes several factors that affect the radar detection effect and makes a detailed summary from the detection environment and other aspects. At the same time, it uses the multisensor system combined with active interference suppression algorithm to design a railway tunnel detection simulation experiment. Experimental results show that the use of multisensors combined with active interference suppression algorithm to optimize radar detection can effectively improve the accuracy of railway tunnel defect detection. Through the analysis of the results of tunnel defect detection, the detection accuracy of this paper has reached 98.8%, which can provide an effective reference for the detection of railway tunnels.

## 1. Introduction

The current railway tunnel construction is a leapfrog development. There are many railway projects in the country under construction. These railways will be the most efficient bridge connecting the country in the future, and the economy will grow rapidly. Therefore, if the construction period is long, on-site construction will often ignore the physical quality of the project. Examples of problems in the operation of railway tunnels are not uncommon in news reports. The lessons are profound, and the results are tragic. Of course, there are many reasons for this tragedy. Everyone involved in the construction is responsible, but in the end, it is due to quality problems. Most of the accidents are caused by the phenomenon of cutting corners and reducing construction procedures during the construction process by the specific construction team at the construction site. At the same time, the competent authority does not supervise such issues nor do a good job of source management that directly affects the quality of the project. It is precisely because many lessons have been learned that the government attaches great importance to the safe operation of railways. This of course puts forward higher requirements for construction quality. The ground penetrating radar method can effectively solve these problems and can guarantee the safety of the railway in operation for future operations.

RETRACTED

There are many methods for tunnel quality inspection. The traditional method is to obtain target information by sampling through boreholes. The detection results obtained by the excavation sampling method are accurate and direct, but only partial information represented by the tunnel lining excavation site can be obtained, and the structure itself has been damaged. Therefore, the quality control of tunnel construction requires an efficient and economical method. It provides continuous detection information without damaging the tunnel lining itself. Since the 1980s, ground penetrating radar detection technology has been expanding its application range due to its fast, nondestructive, and continuous characteristics. However, the complex environmental conditions of the tunnel under construction and many interference sources will affect the effectiveness of radar wave detection at the detection point. Some electromagnetic interference waves generated by these sources directly affect the reflected signal and the waveform of the target body, and it is difficult to remove them in the postprocessing process. In the field test, it should try to avoid these interference sources. Or, it should choose appropriate equipment parameters according to the electromagnetic environment of the construction site to minimize the impact. At the same time, there are other interference factors that affect the accuracy of the detection results, such as environmental humidity, antenna speed, and coupling conditions. The use of ground penetrating radar to comprehensively inspect the tunnel lining structure, finding quality defects and hidden safety hazards and dealing with them in a scientific and timely manner, can avoid serious problems that may even affect the overall safety of the tunnel. It lays a solid foundation for the later completion acceptance and safe operation. It can provide good inspection results and reliable baseline data for project quality evaluation and processing.

In order to overcome active interference, Zhang and Pan proposed an adaptive polarization cancellation method based on dual-polarization radar. They obtain the components and characteristics of the actual target and active interference analysis signal through the vertical and horizontal polarization channels of the dual-polarization radar. Then, in an actual scenario, the weighting factor is subtracted in time to adjust the amplitude and phase difference of the active interference signals received from the two orthogonally polarized channels. This can completely eliminate active interference, but the actual target power will change. In addition, a target signal correction method has been developed to improve the accuracy of monopulse radar angle measurement. Then, through simulation, the factors affecting adaptive polarization cancellation are analyzed in detail. Finally, the experimental results show that it is very effective for the intervention of active blocking and active deception. However, the adaptive method they designed is not flexible enough to meet the actual detection requirements [1]. Zhao et al. researched electronic countermeasures (ECMs) systems to combat misleading electronic countermeasures (ECMs) technology. An adaptive detector uses the generalized probability ratio test (GRLT) standard to detect whether there is any misleading interference in the Fourier transform (FT) field. The proposed detector can analyze initial and auxiliary data through adaptive area echo and misleading interference. Finally, the extended radar network is analyzed as a special case, and the result proves the validity of the digital simulation in the proposed method. However, the scheme they studied is only for special interference [2]. Liu et al. studied the influence of DRFM active jamming technology on coherent pulse compression radar. By introducing the radar signal detection model and radar equation, the influence of the signal generated by DRFM on the detection performance of the radar receiver is analyzed and the relationship between the radar detection probability and the interference power is obtained. Finally, the effective indicators for judging the interference phenomenon are summarized, and the amplitude of the active interference signal is determined. However, their research on the accuracy of radar detection is not deep enough [3]. Yang et al. proposed an error control method based on an active interference suppression control algorithm. It is used to check the parameter uncertainty and noise measurement of the ultrasonic flutter suppression model. The control method can be used to estimate the observed output signal and its time derivative, as well as to model dynamics and measurement noise. Numerical results show that the control method they invented can effectively suppress ultrasonic vibration in the range of large Mach numbers and has obvious adaptability to changes in stiffness parameters. However, the actual suppression effect of the interference suppression algorithm they studied cannot satisfy the research on geology [4]. Chen et al. proposed a new antijamming algorithm based on the minimum mean square error criterion to protect the acquisition stage. The basic idea of the proposed method is the grid search process of sharing synchronization parameters by suppressing interference and receiving signals. The simulation results show that the proposed method can keep the GNSS receiver running during the cold start period with interference signals. In addition, its performance is significantly better than the power reversal method. However, this research method has little meaning for radar detection effect [5]. Yang and Huang studied the interference suppression phenomenon of the integrated coil inductor topology. In the proposed topology, a traditional single-turn spiral inductor is integrated with a built-in tightly coupled LC resonator on the printed circuit board. Interference suppression is achieved by guiding the magnetic flux emitted by the spiral inductor to the tuner instead of other spiral inductors around it. From the experimental results of the comparative case, by changing the value of the coordinator capacitor, the proposed topology can provide design freedom in any frequency band of interest. However, the interference suppression method they proposed is very difficult in practical applications and needs to be simplified [6].

RETRACTED

The innovation of this paper is the use of multiple sensors combined with active interference suppression algorithms to optimize the design of a sensor system for radar defect detection in railway tunnels. It uses a multisensor combination scheme to obtain information such as the angular velocity, acceleration, and magnetic field strength of the carrier. A specific calibration compensation method is selected to calibrate their output values, respectively, which realizes the real-time display of system output data. In this article, an interference suppression algorithm based on Fourier transform is introduced to optimize the interference elements encountered by the radar in the detection of radar. The algorithm first transforms the received data in the Fourier transform fractional domain and then separates the interferometer in the transform domain. By optimizing the design of the gain coefficient, the retention of interference limits is suppressed while signaling time and the frequency response is maximized. Finally, the useful signal after interference suppression is obtained through a short-time inverse Fourier fractional transform. It effectively verifies the effectiveness and simplicity of this method.

RETRACTED

## 2. Multisensor System Combined with Active Interference Suppression Algorithm

### 2.1. The Working Principle of Radar

The essence of radar is an electromagnetic sensor. The basic principle is to send an electromagnetic signal to the area of interest through an antenna [7–9] and judge whether there is a target at the end. At the same time, it receives interesting information such as the distance, radial velocity, angular direction, shape, and bandwidth of the target [10, 11]. The radar system can use this information to perform target detection, ranging, tracking, and imaging functions, as well as the process of determining whether the target exists, that is, radar target detection [12, 13].

Ground penetrating radar (GPR) is generally a method of electromagnetic technology [14, 15]. Compared with other detection methods, the geological radar method can directly see the reflected wave recorded by the radar and can directly analyze the distribution and shape of the structure and target in the tunnel [16, 17]. Combining with the preliminary judgment of the target nature and the detection requirements such as detection depth and minimum resolution, it selects antenna types with different frequencies for the highly selective antenna [18, 19]. The ground penetrating radar will not perform destructive testing on the lining surface, so the same section can be tested repeatedly without damaging the tunnel lining structure. The flexible ground penetrating radar has simple operation, high sampling rate, and fast detection speed. Once the speed and analysis ability reach the centimeter level, it can meet most of the requirements of tunnel structure and target detection, with excellent accuracy [20–22]. Its working principle is shown in Figure 1.

### 2.2. Active Interference Suppression

Active interference suppression generates realistic false signals in the radar's time domain, frequency domain, or image field by emitting interference signals that are very close to the echo signal, which affects the radar's detection of actual targets [23]. For active interference suppression, there are countermeasures from the radar system level and signal processing level [24]. However, most of these methods have active suppression. In order to effectively subdue the active suppression of the radar, it is necessary to study how to detect the active radar to suppress the interference [25].

The biggest difference between suppressive interference and deceptive interference is the degree of interference. It is difficult for the radar to obtain effective echo information because it can fully capture the true time and frequency and convert the echo. If the interceptor is powerful enough, it can completely paralyze the radar, making it impossible to fight against [26]. Active interference suppression mechanisms can be divided into noise amplitude interference, radio frequency noise interference, noise frequency interference, and smart noise interference. According to the implementation strategy of actively suppressing interference, it can be divided into remote support intervention and self-defense intervention [27].  Figure 2 shows the classification of radar interference.

RETRACTED

In the case of passive interference, the radar cannot work normally, mainly because the electromagnetic waves emitted by the radar are reflected or changed through the smoke screen. This kind of interference has a good interference effect, a wide range of influence, low cost, and a wide range of application scenarios. Compared with other types of suppressive interference, the interference effect of noise amplitude interference is smaller and its countermeasures are relatively complete [28]. Noise frequency interference is a new type of interference that mainly affects the chip signal. It can automatically target the center frequency of the radar and has a certain pulse compression gain advantage. In recent years, it has become the focus of interferometer technology research. This study mainly analyzes the differences between different types of interference through the modeling and extraction of feature suppression interference and lays the foundation for subsequent suppression of interference detection and identification.  Figure 3 shows the process of obtaining target information from the radar.

#### 2.2.1. Active Interference Suppression Characteristics

Among the interference factors that affect the radar detection effect, the interference wave generated by the electromagnetic interference object under the action of the electromagnetic field will have a corresponding impact on the radar imaging map. It will cause the imaging spectrum to have no fixed law and range of action. For active interference suppression, extracting its interference characteristics can lay the foundation for radar active interference suppression identification. The following analyzes the six interference patterns to understand their characteristics in the time domain and frequency domain. They extract several characteristic parameters of interference.

*(1) Aiming Frequency Interference.* The time domain expression of noise FM interference is

(1) $$\begin{array}{c} R\left(a\right)=Q_{i}\exp\left[i\left(2\phi f_{i}a+2\phi H_{f_{a}}\int a\left(\varepsilon \right)b\varepsilon +\kappa_{0}\right)\right]. \end{array}$$

Here, *Q*_*i*_ indicates that the magnitude of the interference is a constant, *f*_*i*_ is the carrier frequency that suppresses the interference, and *H*_*fa*_ is the frequency modulation slope of the FM noise.

RETRACTED

The power spectral density of the frequency modulation function *a*(*ε*) can be expressed as follows:

(2) $$\begin{array}{c} H\left(\kappa \right)=\left\{\begin{array}{cc} \frac{\phi_{n}^{2}}{\Delta \kappa }, & 0<\kappa <\Delta \kappa ,\\ 0, & \mathrm{other,} \end{array}\right. \end{array}$$

where Δ*κ* is the modulation bandwidth of the modulation noise *a*(*ε*).

The effective modulation index of the noise FM signal is defined as follows:

(3) $$\begin{array}{c} n_{\kappa e}=\frac{H_{fa}\phi_{n}}{\Delta \kappa }. \end{array}$$

Aiming frequency interference is a kind of noise frequency modulation interference, and its center frequency, interference bandwidth, and effective modulation index generally meet the following conditions:

(4) $$\begin{array}{c} f_{i}=\left(\phi f+f_{0}\right),\\ \Delta \kappa_{i}=\left(2∼5\right)\kappa_{r},\\ n_{fa}<0. \end{array}$$

Here, *f*_0_ represents the center frequency of the radar signal, *ϕf* represents the aiming frequency error, Δ*κ*_*i*_ represents the bandwidth of the aiming interference signal, and *κ*_*r*_ represents the bandwidth of the radar signal. Target frequency interference usually requires that the frequency of the interferometer matches the center frequency of the radar. At the same time, it transmits interference signals with a narrow interference bandwidth, which covers the receiving bandwidth of the radar and requires a high-precision frequency detector to support interference. However, in recent years, with the development of radar frequency flexibility technology, it has become difficult to identify the center frequency of the radar from the interference part and it may be difficult to intercept the target frequency interference on the radar by using frequency interference.

*(2) Blocking Interference.* Blocking interference is a type of FM noise interference. The interference bandwidth and effective configuration index must usually meet the following conditions:

(5) $$\begin{array}{c} f_{i}=\left(\phi f+f_{0}\right),\\ \Delta \kappa_{i}=5\kappa_{r},\\ n_{fa}>0. \end{array}$$

*(3) Sweep Frequency Interference.* Sweep frequency interference can be regarded as a kind of aiming frequency interference whose center frequency is constantly changing. Under normal circumstances, this kind of interference needs to meet the following conditions:

(6) $$\begin{array}{c} \kappa_{i}=\phi f+f_{0}+\frac{\Delta \kappa_{b}}{a}\times A-\frac{\Delta \kappa_{b}}{2}a\in \left[0,a_{b}\right]. \end{array}$$

Here, Δ*κ*_*b*_ is the bandwidth of the frequency sweep interference and *a*_*b*_ is the frequency sweep period of the frequency sweep interference.

RETRACTED

The bandwidth of frequency sweep interference is very large, and it can compete well with flexible-frequency radars and multiple radars of different frequencies. If the given frequency bands are the same, the aggressive interference power will be higher than the cancellation interference power. However, this interference becomes discontinuous in the tie domain after passing through the receiver. The interference scanning frequency represents the number of times a scanning interference scans the entire interference bandwidth per unit time, expressed as follows:

(7) $$\begin{array}{c} \Delta \kappa_{i}=JSF=\frac{1}{A_{b}}. \end{array}$$

Sweep frequency interference will form intermittent pulse interference after passing through the receiver, and the larger the pulse, the denser the pulse.

*(4) Comb Spectrum Interference.* Comb spectrum interference is an interference pattern composed of multiple narrowband interferences, and its expression can be summarized as follows:

(8) $$\begin{array}{c} R\left(a\right)=\sum_{i=1}^{m}R_{i}\left(a\right)+\frac{\Delta \kappa_{a}}{A}\;i=1,2,\ldots ,m, \end{array}$$

where *m* represents the number of narrowband interferences included in the spectrum interference. Each narrowband interference is independent of each other. There are different frequency points in the interference center, and spectrum interference can produce narrowband interference at multiple different frequency points. It can successfully deal with variable frequency radar systems such as flexible-frequency radars and frequency-fluctuation radars.

*(5) Noise Product Interference.* Noise product interference is a new type of interference directed at chirp signals. Its mechanism is to multiply the noise through the filter and the radar pulse signal intercepted by the jammer. This interference can be expressed as follows:

(9) $$\begin{array}{c} R\left(a\right)=m\left(a\right)\times b\left(a\right)\;i=1,2,\ldots ,m, \end{array}$$

where *m*(*a*) is the noise passing through the filter and *b*(*a*) is the chirp signal intercepted by the jammer, and its expression is

(10) $$\begin{array}{c} R\left(a\right)=\text{rect}\left(\frac{1}{A}\right)\exp\left(i2\phi \left(f_{0}+\frac{1}{2}\times \frac{G}{A}a^{2}\right)\right). \end{array}$$

The variable *f*_0_ represents the center frequency of the chirp signal, *G* represents the bandwidth of the FM signal, and A represents the time width of the FM signal. The spectrum of noise product interference can be expressed as follows:

(11) $$\begin{array}{c} I\left(f\right)=M\left(f\right)⊗B\left(f\right). \end{array}$$

*(6) Noise Convolution Interference.* Noise convolution interference is also a new type of interference for chirp signals. Its mechanism is to convolve the noise through the filter with the radar pulse signal intercepted by the jammer. This interference can be expressed as follows:

(12) $$\begin{array}{c} R\left(a\right)=m\left(a\right)⊗B\left(f\right)a>0. \end{array}$$

It can be seen from the representation of the convergence noise interference frequency domain that the convergence noise interference coincides with the center frequency of the transmitting radar signal and the bandwidth is close; that is, the convergence noise interference can be aimed at the center frequency radar. Without precise frequency measurement, it can effectively affect flexible-frequency radars, frequency-differential radars, and other radar systems that allow flexible radar signal ranges. The essence of convergent noise interference can be thought of as amplifying the received chirp signal at different rates and then delaying the addition. Therefore, convergence noise interference can achieve a specific radar pulse compression gain, that is, after the interference is processed by the noise convolutional radar system, it can achieve the same interference effect as other low-power interference suppression.

RETRACTED

### 2.3. Interference Suppression Algorithm

The analysis of active radar interference suppression mainly starts from the feature derivation. Various functional parameters are derived and analyzed from the time domain, frequency domain, and transform domain to lay the foundation for subsequent active radar interference detection. The interference characteristic parameters are as follows.

#### 2.3.1. Frequency-Domain Peak-to-Average Power Ratio after the Receiver

Assuming that the radar echo signal is *v*(*a*), the receiver noise is *d*(*a*) and the received interference is *i*(*a*), then the radar received signal *w*(*a*) can be expressed as follows:

(13) $$\begin{array}{c} w\left(a\right)=v\left(a\right)+d\left(a\right)+i\left(a\right). \end{array}$$

After sampling *w*(*a*), perform the fast Fourier transform to obtain the following:

(14) $$\begin{array}{c} w_{i}\left(n\right)=\frac{w\left(n\right)}{\overset{n}{\underset{n=1}{\max\left(w\left(n\right)\right)}}}\;n=1,2,\ldots ,N. \end{array}$$

The frequency-domain peak-to-average power ratio after the receiver is defined as follows:

(15) $$\begin{array}{c} P_{i}\left(a\right)=10\;\log_{10}\frac{\overset{N}{\underset{n=1}{\max}}w_{i}^{2}\left(n\right)}{1/Nw_{i}^{2}\left(n\right)}. \end{array}$$

The peak-to-average power ratio parameter in the frequency domain mainly reflects the signal variation range in the frequency domain. Its value is relatively high, and the range of comb spectrum interference can be identified by this feature. The flow of the interference suppression algorithm is shown in Figure 4.

RETRACTED

The echo signal is divided into several time periods at equal intervals in the time domain. First, FT is applied to the first time period data, and the optimal order is obtained by searching. By analogy, the optimal order of each time window is obtained. After Fourier transform, the time-frequency aggregation of narrowband and broadband interference is obtained. Then, this is used to detect each time slice. If there is an interference signal, an adaptive gain control method is used to suppress the interference signal to complete the interference suppression.

We calculate the initial value of the argument of *w*(*n*), adopt the principle of the main value interval, and use the optional interval (−*σ* *σ*) as the main value interval to ensure the odd symmetry of the argument with respect to *n* = 0. To eliminate the phase ambiguity of logarithmic changes, there are

(16) $$\begin{array}{c} \ln\left(w\left(a\right)\right)=\ln\left(I\left(a\right)\right)+\ln\left(1+d^{\prime }\left(a\right)\right). \end{array}$$

It can be seen from the formula that the real part and the imaginary part are, respectively,

(17) $$\begin{array}{c} R_{w}\left(a\right)=ie\left[\left(w\left(a\right)\right)\right]=\ln\;W_{i}+ie\left[d^{\prime }\left(a\right)\right],\\ I_{w}\left(a\right)=\ln\left[\ln\;w\left(a\right)\right]=\sigma_{i}+\ln\left[d^{\prime }\left(a\right)\right]. \end{array}$$

Since both the deception interference and the echo signal are zero-average signals, the amplitude of the noise FM interference signal can be estimated as follows:

(18) $$\begin{array}{c} {\hat{W}}_{i}=\exp\left\{\text{mean}\left[R_{w}\left(a\right)\right]\right\}. \end{array}$$

We calculate the interference signal *i*(*a*) from the radar received signal *w*(*a*); then,

(19) $$\begin{array}{c} \hat{d}\left(a\right)=w\left(a\right)-\hat{I}\left(a\right)\\ =d^{\prime }\left(a\right)+I\left(a\right)\left[1-\frac{{\hat{W}}_{i}}{{\hat{W}}_{i}}\exp\left(iIn\left(d^{\prime }\left(a\right)\right)\right)\right]. \end{array}$$

## 3. Experiment of Railway Tunnel Radar with the Multisensor System Combined with Active Interference Suppression Algorithm

As a kind of concealed project, tunnel construction will inevitably have defects in the construction process. Due to its concealment, defect detection has become a concern of tunnel workers. Geological radar detection is a fast and efficient detection method. Its principle is the same as that of the tunnel lining structure. The tunnel lining structure is combined with radar detection for tracking tunnel defects.

RETRACTED

The ground penetrating radar is used for nondestructive testing of tunnel lining, and its main purpose is to ensure that the construction quality of tunnel lining meets the requirements of design specifications. The tested elements are the initial support, secondary lining and inverted arch, concrete thickness detector, double-layer secondary lining thickness, gaps and nonsolid areas, and concrete compression of the backfill layer.

Due to the unevenness of the coated concrete, when the electromagnetic wave propagates to the initial support and the secondary coating, the speed of the electromagnetic wave will change within a certain range. We need to adjust the parameters of the medium to be measured on the concrete. If we want to calibrate the relative permeability or electromagnetic velocity of shotcrete before the first support material inspection, we can use the core perforation sampling method to calibrate three or more positions and take the average value. In this paper, the tunnel is inspected in the part where the concrete thickness is known, because the core drilling sampling method will damage the back wall to calibrate the parameters of the secondary cladding concrete. The parameters of the radar include the number of sampling points, sampling rate, and band-pass filtering. The number of sampling points represents the number of sampling points in each acquisition dataset. This article sets the number of sampling points to 400. In order to make the recorded waveform more complete and controllable, the sampling rate is selected to be 6 times the antenna center frequency. In the processing of data and interference waves, band-pass filtering is used.

Due to the requirement of a safe step between the surface and cladding of the tunnel under construction, the construction of the tunnel cladding should be monitored quickly. Therefore, the initial support inspection should monitor the construction progress. It should take into account the inspection progress, that is, whether the age of the concrete can meet the inspection requirements. Before the inspection, the side walls of the cladding should be clearly marked with red paint every 5 meters, indicating the number of kilometers and the number of piles. If necessary, the detection location should be clearly marked to ensure the accuracy of the detection data.

The main control measures for the secondary cladding inspection of the tunnel are used for cavities, defects, cladding thickness, inverted thickness, filler layer and other cladding, the distribution of steel bars in the cladding, and the solid lining of the initial support. The main detection method is the geological radar method. The tunnel wall inspection is to place inspection lines on the tunnel warehouse, the center arch on both sides, the side walls, and the inverted arch on both sides. Or, it provides a basic overview of the cross section of the intersection. And, it focuses on the encrypted overview of specific tunnel sections or irregularly covered structural sections, as well as gives the basic knowledge of paving leaks, horizon cracks, and crevices.  Figure 5 is a schematic diagram of radar defect detection in railway tunnels.

RETRACTED

The tunnel defect detection system requires methane sensors, temperature and humidity sensors, wind speed and direction sensors, noise sensors, brightness detectors, and air pressure detectors. At the same time, it cooperates with radar to detect railway tunnels. And, it provides statistics on the size and location of defects behind the tunnel lining and summarizes the distribution of specific types of defects. The defect classification table is now introduced.  Table 1 is the tunnel defect classification table.

In the detection of railway tunnel defects, firstly, the relevant sensors in the defect detection system are used to obtain the data related to the tunnel defects at the moment and then the output data of the sensors are processed accordingly. In this process, any calculation processing is based on sensor data. Therefore, the sensor plays a vital role in the tunnel defect detection system. Different sensors have different test principles and applicable conditions. These will affect the results of tunnel defect detection and the application environment of the system.  Figure 6 is the design of a multisensor system for railway tunnel defect detection.

The noise sensor, temperature and humidity sensor, wind speed and direction sensor, and methane sensor are combined with a high-precision microprocessor as the control and calculation unit to obtain the relevant information of the railway tunnel and obtain the environmental factors of the tunnel. Then, it cooperates with the air pressure detector, light brightness detector, and magnetic field detector to obtain the air pressure, light brightness, and magnetic field strength in the tunnel.

## 4. Experimental Results and Analysis

### 4.1. Simulation Analysis of the Multisensor System Combined with Active Interference Suppression Algorithm

In order to analyze the algorithm more deeply, simulation experiments are carried out using the algorithm.  Figure 7 is a histogram of phase statistics. It can be seen from the figure that the echo is widely distributed in the entire phase interval, and the echo and interference have obvious different phase distribution characteristics. In contrast, the interference is only concentrated on a limited phase. Therefore, the interference and echo can be identified through the conventional discrimination model of the tree.

RETRACTED

Figure 8 shows the output waveforms of the radar-matched filter before and after interference suppression. It can be seen from Figure 8(a) that before the interference suppression of the matched filter, both the target and the interference spike exist in its output. Therefore, the radar cannot achieve the purpose of extracting real target information by selecting target spikes from multiple spikes. In contrast, the matched filter output in Figure 8(b) has only a target spike after interference suppression, and the radar can extract the distance information of the real target through this spike.

Figure 9 is a performance graph of the radar suppression algorithm. Under various conditions, the target echo similarity curve is consistent with the probability curve of correct target recognition after radar interference. It can be seen from this figure that as the signal-to-noise ratio increases, the interference and echo similarity coefficient increases. And, the phase is sensitive to the influence of noise under low signal-to-noise ratio, and it is not easy to be distinguished.

Figure 10 is the comparison result of several methods under different frequency deviations. It can be seen from the figure that when the frequency estimation performance of the improved method reaches the optimum, the frequency deviation in the constraint condition can be satisfied. At this time, the frequency estimation accuracy of the improved method is significantly higher than that of the other three methods.

### 4.2. Defect Detection Problems in Railway Tunnels

As an important nondestructive testing method, radar has been accepted by engineers. At present, it is widely used in the inspection of heavy and large projects at home and abroad, and it controls the quality of the project very well. However, due to various factors, there are more or less problems in the application of geological radar. In response to these problems, the application scholars of the ground penetrating radar have done a lot of research in order to reduce the detection error of the ground penetrating radar. This article specifically studies and analyzes tunnel lining inspection and lists the factors that affect tunnel inspection, so as to improve the accuracy of domestic tunnel lining inspection. It provides safety guarantee for tunnel engineering.

Concrete is a relatively stable synthetic material. It is a nonelectric good conductor, that is, a nonconductive substance. From Table 2, we can see that the dielectric properties of concrete will also have an impact due to the difference in water content.

RETRACTED

As shown in Figure 11, according to the dielectric constant results of concrete at different ages, the dielectric constant of concrete at 3d, 7d, 14d, and 28d age was analyzed.

In addition to the relative permittivity and permeability of the medium, the vertical resolution of the ground penetrating radar is also related to the center frequency of the antenna. When the medium is constant, the vertical resolution of the ground penetrating radar is inversely proportional to the center frequency of the radar antenna. Regarding the influencing factors, radar should pay attention to the selection of detection timing when detecting defects. At the same time, when facing electromagnetic interference, it should be far away from these interference sources or appropriate shielding measures should be selected to minimize the impact.

### 4.3. The Detection Results of Railway Tunnel Radar Optimization

In the process of detecting defects in railway tunnels, electromagnetic waves first pass through the air medium and enter the concrete medium. For air and concrete media, the reflection coefficient is negative. In other words, electromagnetic waves are negative. Therefore, the first wave of the measurement results is inconsistent and the difference is large.  Table 3 shows the measurement location information of the first wave.

Figure 12 is the detection accuracy and error analysis results of the railway tunnel radar defect detection of the multisensor system combined with active jamming algorithm.

It can be seen from the figure that the traditional detection method can easily make the cladding thickness too large or too small, resulting in a large error of up to 0.042 m in the identification and evaluation of railway tunnel defects. It greatly reduces the reliability and is easy to make wrong estimates or cause unnecessary losses. The detection method optimized by combining multiple sensors and active interference suppression algorithm can confirm that the error is within 0.02 m. The multisensor defect detection rate combined with the active interference suppression algorithm is 98.8%, which can effectively improve the detection accuracy.

## 5. Conclusion

In this paper, the defect detection of railway tunnels is optimized with the multisensor system combined with active interference suppression algorithm and a related sensor detection system is designed. The multisensor detection system includes temperature and humidity sensors, wind speed and direction sensors, methane sensors, and noise sensors. It can meet the needs of tunnel curve detection, and the multisensor detection system has higher stability and accuracy. It starts from the basic principles of ground penetrating radar and electromagnetic field theory, according to the propagation characteristics and laws of electromagnetic waves and various tunnel radar detection parameters and indicators, to study data acquisition, processing, and transmission methods. The results of radar detection factors of railway tunnels include the influence of equipment parameters and the influence of the external detection environment. In this paper, combined with relevant examples of mechanical substance detection, the specific application of ground penetrating radar in various factors that affect the quality of tunnel detection, matters needing attention, railway tunnel radar detection, etc., is analyzed. It focuses on analyzing the amplitude and polarity of the reflected wave, the spectral characteristics of the reflected wave, the morphological characteristics of the internal axis of the reflected wave, and the influence of interference waves. At the same time, this paper studies the influence of water and air on the dielectric constant of concrete and the influence of various factors on the radar detection, such as the choice of detection timing when detecting the thickness of concrete. Finally, it is hoped that the content studied in this article can provide useful information and reference value for radar operators.

RETRACTED

## Figures and Tables

**Figure 1:** Radar working principle diagram.

**Figure 2:** Radar jamming classification.

**Figure 3:** The process of radar acquiring target information.

**Figure 4:** Flow chart of interference suppression algorithm.

**Figure 5:** Schematic diagram of railway tunnel radar defect detection.

**Figure 6:** Design of the multisensor system for railway tunnel detection.

**Figure 7:** Source signal phase statistics histogram.

**Figure 8:** Radar-matched filter output waveform (a) before and (b) after interference suppression.

**Figure 9:** Radar suppression algorithm performance graph.

**Figure 10:** Comparison results of several methods under different frequency deviations.

**Figure 11:** The lining thickness of concrete of different ages.

**Figure 12:** Detection accuracy and error.

**Table 1:** Tunnel defect classification table.

Defective item	Defect level	I	II	III	IV
		Slight defect length (m)	More serious defect length (m)	Severe defect length (m)	Very serious defect length (m)

There is a cavity behind the lining	There is a hole	≤1	1 ≤ *L* ≤ 3	3 ≤ *L* ≤ 5	>5
Backfill is not dense	Not dense	≤3	3 ≤ *L* ≤ 9	9 ≤ *L* ≤ 15	>15
The base is not dense	Not dense	≤3	3 ≤ *L* ≤ 9	9 ≤ *L* ≤ 15	>15

RETRACTED

**Table 2:** The difference between the dielectric constant of each parameter and the thickness of the test.

Dielectric constant		Volume ratio%		Concrete dielectric constant	Calculated lining thickness
Air	Water	Air	Water		

1	81	5	1	6.25	0.38
1	81	4	2	6.74	0.37
1	81	3	3	7.32	0.36
1	81	2	4	7.68	0.35
1	81	1	5	8.31	0.34

**Table 3:** First wave signal position table.

Number	First wave signal position (ns)	Mean difference (ns)	Maximum difference (ns)	Minimum difference (ns)

1	3.9	−0.23	0.22	−0.18
2	3	0.09	0.28	−0.32
3	3.16	0.17	0.16	−0.11
4	3.18	0.14	0.14	−0.11
5	3.71	0.09	0.13	−0.16
6	3.83	−0.12	0.22	−0.05
7	3.34	−0.17	0.07	−0.24
8	3.83	0.27	0.19	−0.11
9	3.66	0.18	0.11	−0.15
10	3.78	0.21	0.14	−0.12

## Data Availability

The data used to support the findings of this study are available from the corresponding author upon request.
